This article has been retracted.

# Analysis of Risk Factors of Bronchiolitis Obliterans in Children with Mycoplasma pneumoniae Bronchiolitis

**DOI:** 10.1155/2022/9371406

**Published:** 2022-03-01

**Authors:** KunLing Huang, Jianhua Liu, Wenshan Lv, Yajuan Chu, Baochi Li, Peng Wu, Jinfeng Shuai

**Affiliations:** Respiratory Department II, Hebei Children's Hospital, No. 133 Jianhua South Street, Shijiazhuang, 050031 Hebei, China

## Abstract

**Objective:**

To investigate the related risk factors for bronchiolitis obliterans (BO) in children with mycoplasma pneumonia (MP) bronchiolitis.

**Method:**

The clinical data of 227 children with MP bronchiolitis who were admitted to the II Department of Respiratory of Children's Hospital of Hebei Province from January 2018 to June 2020 were retrospectively analyzed. According to the sequelae of BO, they were divided into 32 cases in the BO group and 195 cases in the non-BO group. The univariate analysis was performed on the clinical and laboratory parameters of the two groups, and the multifactor logistic regression was performed further to determine the independent risk factors for the occurrence of BO in MP bronchiolitis, and then, the cut-off value with the maximum diagnostic value of indicators was found through the ROC curve analysis.

**Results:**

The results of univariate and multivariate logistic regression analysis showed that the independent risk factors for the occurrence of BO in MP bronchioles were longer duration of moist rales (OR = 1.203, *P* = 0.003), higher levels of serum lactate dehydrogenase (LDH) (OR = 1.005, *P* = 0.036), hypoxemia (OR = 7.442, *P* = 0.035), and pleural effusion (OR = 4.437, *P* = 0.004). The area under the ROC curve was 78.2%, 72.0%, 68.2%, and 71.0%, respectively (*P* < 0.001). The cut-off value of duration of moist rales and levels of serum LDH are 7.5 d and 330 U/L, respectively.

**Conclusion:**

Children with MP bronchiolitis with high serum LDH level (≥330 U/L), combined with hypoxemia, pleural effusion, and lung wet rale duration (≥7.5 d), may be more prone to BO, in which lung wet rale duration prediction value is the largest. Among them, duration of pulmonary moist rales has the highest predictive value.

## 1. Introduction

Bronchiolitis obliterans (BO), also known as constrictive bronchiolitis, is a rare small airway chronic obstructive pulmonary disease, which is bronchiole stenosis or/and occlusion caused by fibrosis around the bronchioles and submucosa [1]; it can be caused by infection, organ or stem cell transplantation, inhalation of toxic substances, autoimmune diseases, and gastroesophageal reflux [2–5]. Most of the pathogens are viruses, and adenovirus infection is the most common [6]. MP is one of the common pathogens of respiratory tract infections in children. In recent years, the BO caused by MP infection has gradually increased, and it is also a common pathogen of BO after infection [7, 8]. MP infection can cause bronchiolitis, lobar pneumonia, bronchopneumonia, and other different manifestations, resulting in different types of pneumonia; clinical features and prognosis are different. BO after MP infection is mostly secondary to acute bronchiolitis [7, 9]. However, there are few studies on the incidence and risk factors of BO after MP bronchiolitis, partly due to the limited number of patients [10]. With the increase of BO in children with MP bronchiolitis, most of the children with BO are characterized by recurrent cough and asthma, poor exercise endurance, recurrent respiratory tract infection, and impaired lung function. Serious cases need long-term family oxygen therapy, which affects the quality of life and even endangers the lives of children [11]. The poor prognosis of BO after infection is related to the delayed diagnosis and the formation of pulmonary fibrosis. Therefore, early identification of the risk factors for the occurrence of BO in MP bronchiolitis and early intervention are of great significance to reduce the occurrence of BO and improve the prognosis of children. This study retrospectively analyzed the hospitalized medical records of 32 children with BO and 195 children without BO after MP bronchiolitis, aiming to find high-risk factors for BO in MP bronchiole.

## 2. Objectives and Methods

### 2.1. Research Object

A total of 227 children with MP bronchiolitis hospitalized in the Respiratory Department of Hebei Children's Hospital from January 2018 to June 2020 were included, including 136 males and 91 females. The patients were followed up for at least half a year after discharge. According to the sequelae of BO, the patients were divided into a study group (*n* = 32) and control group (*n* = 195) without BO. The study was approved by the Hospital Ethics Committee (Medical Research Ethics Committee No. 212), and informed consent was signed by parents.

### 2.2. Inclusion and Exclusion Criteria

#### 2.2.1. Inclusion Criteria

1. Age from 1 month to 18 years old
2. All the children met the diagnostic criteria of MP bronchiolitis [12, 13]: (1) there are clinical manifestations of acute infection such as cough and fever. Chest CT examination showed unilateral or bilateral tree bud sign, central lobular nodule, bronchiolitis, and other bronchiolitis; (2) use gelatin particle agglutination test to detect serum MP antibody (mixed antibody of IgM and IgG) titer and single MP antibody titer ≥1 : 160 or compare the recovery period, and the acute-phase MP antibody titer is 4 times or more than 4 times higher or reduced
3. Diagnostic criteria for BO in the study group refer to “diagnosis and treatment of bronchiolitis obliterans in children” [14]

#### 2.2.2. Exclusion Criteria

1. Children with incomplete case data
2. Children lost to follow-up
3. Children with basic diseases such as chronic lung disease or low immune function
4. The child was diagnosed with BO before this illness
5. Combined organ or stem cell transplantation, autoimmune diseases, and other causes can cause BO in children

### 2.3. Research Methods

The medical records of children with MP bronchiolitis during hospitalization were collected retrospectively: (1) general information such as gender and age; (2) clinical manifestations (symptoms and signs); (3) lung imaging (type and location of lesions); (4) laboratory indicators such as peripheral blood white blood cells (WBC), C-reactive protein (CRP), lactate dehydrogenase (LDH), etc. within 24 hours of admission; (5) mixed infections (multiple pathogen detection of sputum and respiratory tract, sputum and alveolar lavage fluid culture, double-site blood culture, etc. detected viruses or bacteria and other pathogens); (6) intrapulmonary and extrapulmonary complications; (7) bronchoscopic manifestations (children with bronchoscopy indications, parents signed informed consent, underwent bronchoscopy and bronchoalveolar lavage, and observed bronchoscopy manifestations); and (8) treatment (glucocorticoids and noninvasive CPAP-assisted ventilation).

### 2.4. Statistical Processing

SPSS25.0 software was used for statistical analysis. The measurement data were skewed distribution, expressed by median (quartile distance) *M* (P25-P75), and Mann–Whitney *U* test was used for comparison between groups. The enumeration data were represented by the number of cases (percentage) *n* (%), and the comparison between groups was performed by the *χ*^2^ test or continuous correction of *χ*^2^ value or Fisher exact probability method. Multivariate logistic regression analysis was performed on statistically significant variables between the two groups. *P* < 0.05 indicated that the difference was statistically significant.

## 3. Result

In general, there were 32 cases in the BO group, including 24 males and 8 females, aged from 1 to 14 years old, and 195 patients in the non-BO group, including 112 males and 83 females, aged from 1 to 10 years old. The incidence of BO after MP bronchiolitis was 14%. There was no significant difference in sex and age between the two groups (*P* > 0.05), as shown in Table 1.

### 3.1. Comparison of Clinical Data of Two Groups of Children

The number of involved lobes (≥4), bronchoscopic mucus thrombus, and noninvasive CPAP application in the BO group were higher than those in the non-BO group. The duration of wet rale in the BO group was longer than that in the non-BO group, and the difference was statistically significant (*P* < 0.05), as shown in Table 1.

### 3.2. Etiological Examination Results

In the BO group, bacteria were detected in 4 cases (12.5%), including 1 case of Streptococcus pneumoniae, 1 case of Klebsiella pneumoniae, 1 case of Moraxella catarrhalis, and 1 case of Staphylococcus aureus; virus was detected in 4 cases (12.5%), including 1 case of respiratory syncytial virus, 1 case of adenovirus, and 1 case of influenza A virus. Bacteria were detected in 14 children (7.2%) in the non-BO group, including 5 cases of Streptococcus pneumoniae, 3 cases of Klebsiella pneumoniae, 3 cases of Moraxella catarrhalis, 2 cases of Staphylococcus aureus, and 1 case of Escherichia coli. The virus was detected in 30 cases (15.4%), including 9 cases of respiratory syncytial virus, 6 cases of adenovirus, 5 cases of influenza A virus, 4 cases of influenza B virus, 3 cases of parainfluenza virus, and 3 cases of coronavirus, nasal. There were 2 cases each of virus and metapneumovirus, and 4 cases were infected with both viruses. There was no significant difference in mixed bacterial and viral infections between the two groups of children (*P* > 0.05), as shown in Table 1.

### 3.3. Comparison of Laboratory Indexes between Two Groups of Children

The level of serum LDH in the BO group was significantly higher than that in non-BO group, and the difference was statistically significant (see Table 2).

### 3.4. Multivariate Logistic Regression Analysis of BO Risk Factors after MP Bronchiolitis

With BO as the dependent variable, hypoxemia, pleural effusion, the number of lesions involved (≥4), mucus embolism under bronchoscopy, noninvasive CPAP-assisted ventilation, duration of moist rales, and serum LDH level were statistically significant in the two groups. The forward stepping (conditional) method was used for multivariate logistic regression analysis. The results showed that hypoxemia, LDH, pleural effusion, and duration of moist rales were the risk factors for the occurrence of BO in MP bronchiolitis (*P* < 0.05), as shown in Table 3.

### 3.5. ROC Curve of BO Risk Factors after MP Bronchiolitis

ROC curves were plotted for the risk factors (duration of moist rales, LDH, hypoxemia, pleural effusion, and so on) of BO in MP bronchiolitis (see Figure 1). The areas under the ROC curves were 78.2%, 72.0%, 68.2%, and 71.0%, respectively (all *P* values were less than 0.001). The area under the ROC curve of duration of moist rales was the largest; that is, the predictive value of BO after MP bronchiolitis was the largest. The critical values of wet rale duration and LDH for predicting BO after MP bronchiolitis were 7.5 d (sensitivity 78.1%, specificity 64.6%) and 330 U/L (sensitivity 59.4%, specificity 76.4%), respectively.

## 4. Discussion

BO is a rare and serious chronic obstructive pulmonary disease. The main mechanism is airway epithelial cell injury and subsequent fibroblast proliferation. In children, BO is the most common after infection. Adenovirus is the most common cause of BO after infection in children. MP is the second cause of BO after adenovirus. MP infection of the respiratory tract can promote local immune response and cause airway epithelial cell damage, shedding, and granulation tissue hyperplasia. Current studies suggest that [7, 9] MP-related BO may occur after acute bronchiolitis. The lung biopsy results of a 17-year-old case [15] and Rollins et al. and other studies [16] support this theory. In this study, 227 children with MP bronchiolitis were followed up for half a year. 32 cases (14%) had relatively high prevalence of BO after MP bronchiolitis, which may be partly related to the selected cases of MP acute bronchiolitis. The incidence of BO caused by adenovirus infection ranges from 1.7% to 47.4%, with a large difference [17–19]. At present, there is a lack of multicenter, large sample studies on the prevalence and risk factors of BO after MP pneumonia. The results of this study showed that hypoxemia, pleural effusion, high serum LDH level, and duration of moist rales were independent risk factors for BO after MP bronchiolitis. Among them, the area under ROC curve of duration of moist rales in the lung was the largest, and the prediction value for BO was the largest. This study provides a possible theoretical basis for the clinical prevention of BO after MP infection.

In the cases of BO after adenovirus infection, some studies have shown that invasive mechanical ventilation is a risk factor for the occurrence of BO [18, 19], and some studies have suggested that hypoxemia is a risk factor for the occurrence of BO [20]. In this study, 227 cases of bronchiolitis were not treated with invasive mechanical ventilation, but 8 cases (28.0%) were treated with noninvasive CPAP, which was significantly higher than that in the group without BO (1.0%). The difference was statistically significant, but it was not an independent risk factor for BO. In our study, hypoxemia is a risk factor for BO in MP bronchiolitis, which is consistent with the research results of Wen et al. [9] on the occurrence of BO in MP bronchiolitis and hypoxemia. MP bronchiolitis is mainly bronchiolitis, which can be complicated with atmospheric tract inflammation, such as epithelial cell injury, mucosal barrier destruction, inflammatory cell infiltration, lumen inflammatory exudation and necrotic tissue, lumen fibrosis, airway distortion, and even occlusion [21]. Patients with mild MP bronchiolitis showed fever and cough, and some are accompanied by wheezing. Patients with severe lesions had large and small airway smooth muscle spasm and secretion obstruction and hypoxemia. Noninvasive CPAP-assisted ventilation or mechanical ventilation was needed [12]. If hypoxia cannot be corrected in time, it can further aggravate airway inflammation, aggravate lung damage, and even cause irreversible lung damage, thereby promoting the occurrence of BO.

The persistent moist rales and wheezing sounds can be heard in the lungs of children with BO. In this study, there was no significant difference in the incidence of moist rales and wheezing sounds between the two groups, but the duration of moist rales in the BO group was significantly longer than that in the non-BO group, and the difference was statistically significant, indicating that the duration of moist rales was long, which could promote the occurrence of BO after MP bronchiolitis. The occurrence of moist rales in children with MP bronchiolitis is related to small airway inflammation, intracavitary exudation, or granulation tissue formation after MP infection [21]. Bronchiolitis persists after MP infection. Exudates, necrotic tissue, and granulation tissue block the lumen, resulting in bronchial lumen stenosis. Some children have moist rales or wheezing sounds. With the improvement of inflammation, rales disappear. For example, inflammation continues to progress, and tissue fibrosis around the small airway and the formation of granulation tissue in the lumen continue to lead to bronchial lumen stenosis, destruction, or even occlusion and ultimately develop into BO. The moist rale is a clinical manifestation of BO, and the persistence of moist rale may suggest that MP bronchiolitis develops into BO.

Pleural effusion is one of the common pulmonary complications of MP pneumonia. MP infection can lead to pleural inflammation; increased effusion; release of various enzymes, complements, bioactive substances, and inflammatory immune response; and promote the formation of pleural effusion. MP pneumonia with pleural effusion had longer fever, higher inflammatory indexes and biochemical indexes, stronger systemic inflammatory response, and heavier airway injury [22]. Pleural effusion is one of the clinical manifestations of severe MP pneumonia. Studies have shown that [23] severe pneumonia is a risk factor for BO after MP pneumonia. In this study, 20 cases (62.5%) of the BO group were complicated with pleural effusion, accompanied by elevated lactate dehydrogenase, which was severe pneumonia, suggesting that strong inflammatory response may promote the occurrence of BO, indicating that pleural effusion is an independent risk factor for BO after MP bronchiolitis.

LDH is a glycolytic enzyme, which is widely distributed in the cytoplasm of the skeletal muscle, liver, heart, and other important organs. When the cell membrane is destroyed or the cell is dissolved, the intracellular LDH is released into the blood, resulting in an increase in the level of LDH in the serum. When MP infected the body, airway and lung tissue cells were destroyed, LDH can be released into the extracellular, and serum LDH content increased. Therefore, LDH is one of the related inflammatory indicators of infection, and the level of serum LDH is an independent predictor of refractory MP pneumonia in children. To a certain extent, it can reflect the clinical severity of the disease, and it is also one of the indicators to predict the prognosis of patients with community-acquired pneumonia [24, 25]. This study suggests that higher levels of serum LDH are related to the increased risk of BO in children with MP bronchiolitis, which is consistent with the findings of Atag et al. [10] that serum LDH level is an independent risk factor for BO in MP pneumonia.

In summary, BO is not uncommon after MP pneumonia. When children have MP bronchiolitis and high serum LDH level (≥330 U/L), combined with hypoxemia, pleural effusion, and long duration of pulmonary rales (≥7.5 d), they should be highly alert to the occurrence of BO after infection, regular clinical follow-up, early diagnosis, and treatment, which can improve the quality of life of children with BO. This study has certain limitations. First of all, the gold standard of BO diagnosis is lung biopsy, but it is an invasive method. The diagnosis in this paper is based on chest high-resolution lung CT and clinical features. Secondly, this study is a single-center and retrospective study, which may not include all the observation indicators related to BO occurrence. In the future, multicenter and prospective studies can be carried out on the risk factors of BO in MP bronchiolitis.

## Figures and Tables

**Figure 1:** ROC curve of BO risk factors after MP bronchiolitis.

**Table 1:** Comparison of clinical data of two groups of children.

Clinical indicators	BO group (32 cases)	Group without BO (195 cases)	Statistics (*χ*^2^*/Z/-*)	*P* value
General information				
Gender (male/female)	24/8	112/83	3.531	0.060
Age (years)	5 (3-6)	5 (3-7)	-0.57	0.569
Time from onset to application of macrolides (d)	4 (3-5)	3 (3-5)	-1.630	0.103
Family or personal allergy history (case)	16 (50.0%)	116 (59.5%)	1.017	0.313
Symptoms and signs				
Fever (case)	28 (87.5%)	186 (95.4%)	1.873	0.171
Hot peak (°C)	39.6 (38.9-40)	39.3 (39.0-39.8)	-0.150	0.881
Heat path (d)	8.5 (6.0-10.0)	8 (7-10)	-0.815	0.415
Respite (case)	7 (21.9%)	26 (13.3%)	1.000	0.317
Shortness of breath (case)	4 (12.5%)	8 (4.1%)	2.376	0.123
Hypoxemia (case)	12 (37.5%)	2 (1.0%)	57.049	≤0.001
Moist rales (case)	32 (100%)	174 (89.2%)	2.623	0.105
Duration of moist rales (d)	10.5 (8.0-13.0)	6 (4-8)	-5.127	≤0.001
Iconography				
Pleural effusion (case)	20 (62.5%)	40 (20.5%)	24.922	≤0.001
Small consolidation (case)	8 (25.0%)	73 (37.4%)	1.852	0.174
Lesion site (double/single)	24/8	118/77	2.463	0.117
Number of lesions involving leaves (1)	1 (3.1%)	21 (10.8%)	1.835	0.176
Number of lesions involving leaves (2)	8 (25.0%)	76 (39.0%)	2.303	0.129
Number of lesions involving leaves (3)	4 (12.5%)	55 (28.2%)	3.525	0.060
Number of lesions involving leaves (≥4)	19 (59.4%)	43 (22.0%)	19.289	≤0.001
Coinfection				
Bacteria (case)	4 (12.5%)	14 (7.2%)	0.462	0.497
Virus (case)	4 (12.5%)	30 (15.4%)	0.025	0.876
Extrapulmonary complications (case)	6 (18.8%)	29 (19.0%)	0.001	0.979
Skin lesion (case)	1 (3.1%)	2 (1.0%)	—	0.367
Functional disturbance of the gastrointestinal tract (case)	0	5 (2.6%)	—	1.000
Electrolyte disturbance (case)	0	3 (1.5%)	—	1.000
Hepatic dysfunction (case)	6 (18.8%)	24 (12.3%)	0.512	0.474
Myocardial damage (case)	4 (12.5%)	20 (10.3%)	0.005	0.942
MP titer			0.871	0.832
1 : 160	1 (3.1%)	8 (4.1%)		
1 : 320	3 (9.4%)	19 (9.7%)		
1 : 640	4 (12.5%)	15 (7.7%)		
1 : 1280	24 (75%)	153 (78.5%)		
Treatment				
Bronchoscope (case)	21 (65.6%)	105 (53.8%)	1.544	0.214
Microscopic appearance: mucus plug (case)	12 (37.5%)	11 (5.6%)	27.243	≤0.001
Hormone application (case)	24 (75.0%)	129 (66.2%)	0.979	0.322
Time from onset to application of hormones (d)	11 (10-12)	10 (8.5-13.0)	-0.778	0.437
Application of noninvasive CPAP (case)	8 (25.0%)	2 (1.0%)	32.041	≤0.001

**Table 2:** Comparison of laboratory indexes between two groups of children.

Laboratory index	BO group (32 cases)	Unretained BO group (195 cases)	Statistics (*Z*)	*P* value
WBC (×10^9^/L)	8.5 (8.0-13.0)	8.2 (6.4-10.1)	-1.577	0.115
Neutrophil percentage (%)	63.6 (56.2-65.9)	61.2 (52.3-67.7)	-0.305	0.760
CRP (mg/L)	15.5 (6.0-38.0)	10.0 (6.0-18.0)	-1.664	0.096
Percentage of eosinophils (%)	1.55 (1.13-2.08)	1.10 (0.50-2.50)	-1.461	0.144
Erythrocyte sedimentation rate (mm/h)	29.5 (19.3-46.5)	23.0 (16.0-39.3)	-1.688	0.091
LDH (U/L)	334.5 (281.3-510.0)	276.0 (250.0-327.0)	-3.987	≤0.001
D-dimer(mg/L)	1.12 (0.38-2.02)	0.79 (0.47-1.28)	-1.000	0.307

**Table 3:** Multivariate logistic regression analysis results of BO risk factors.

Risk factors	Regression coefficient	Standard error	*P* value	OR	95% CI
Hypoxemia	2.007	0.953	0.035	7.442	1.148-48.225
LDH	0.005	0.002	0.036	1.005	1.000-1.009
Hydrothorax	1.490	0.515	0.004	4.437	1.616-12.181
Duration of moist rales	0.185	0.062	0.003	1.203	1.066-1.358
Constant	-5.713	0.989	≤0.001	0.049	

## Data Availability

No data were used to support this study.
